This article has been retracted.

# Oral supplementation of diabetic mice with propolis restores the proliferation capacity and chemotaxis of B and T lymphocytes towards CCL21 and CXCL12 by modulating the lipid profile, the pro-inflammatory cytokine levels and oxidative stress

**DOI:** 10.1186/s12865-015-0117-9

**Published:** 2015-09-15

**Authors:** Ahmad A. Al Ghamdi, Gamal Badr, Wael N. Hozzein, Ahmed Allam, Noori S. Al-Waili, Mohammed A. Al-Wadaan, Olivier Garraud

**Affiliations:** Chair of Engineer Abdullah Baqshan for Bee Research, College of Food and Agriculture Sciences, King Saud University, Riyadh, Saudi Arabia; Laboratory of Immunology and Molecular Physiology, Zoology Department, Faculty of Science, Assiut University, Assiut, 71516 Egypt; Bioproducts Research Chair, Department of Zoology, College of Science, King Saud University, Riyadh, Saudi Arabia; Botany Department, Faculty of Science, Beni-Suef University, Beni-Suef, Egypt; Zoology Department, Faculty of Science, Beni-Suef University, Beni-Suef, Egypt; Al-Waili’s Foundation for Science, New York, USA; Institut National de la Transfusion Sanguine, Paris, Université de Lyon, Saint-Etienne, France

## Abstract

**Background:**

Type 1 diabetes mellitus (T1D) is a chronic autoimmune disease caused by the selective destruction of pancreatic β cells, followed by hyperglycemia, oxidative stress and the subsequent extensive impairment of immune cell functions, a phenomenon responsible for the development of chronic diabetic complications. Propolis, a natural bee product that is extensively used in foods and beverages, significantly benefits human health. Specifically, propolis exerts antioxidant, anti-inflammatory and analgesic effects that may improve diabetic complications. To further elucidate the potential benefits of propolis, the present study investigated the effect of dietary supplementation with propolis on the plasma cytokine profiles, free radical levels, lipid profile and lymphocyte proliferation and chemotaxis in a streptozotocin (STZ)-induced type I diabetic mouse model.

**Methods:**

Thirty male mice were equally distributed into 3 experimental groups: group 1, non-diabetic control mice; group 2, diabetic mice; and group 3, diabetic mice supplemented daily with an ethanol-soluble derivative of propolis (100 mg/kg body weight) for 1 month.

**Results:**

First, the induction of diabetes in mice was associated with hyperglycemia and significant decreases in the insulin level and the lymphocyte count. In this context, diabetic mice exhibited severe diabetic complications, as demonstrated by a significant decrease in the levels of IL-2, IL-4 and IL-7, prolonged elevation of the levels of pro-inflammatory cytokines (IL-1β, IL-6 and TNF-α) and reactive oxygen species (ROS) and altered lipid profiles compared with control non-diabetic mice. Moreover, antigen stimulation of B and T lymphocytes markedly reduced the proliferative capacity and chemotaxis of these cells towards CCL21 and CXCL12 in diabetic mice compared with control mice. Interestingly, compared with diabetes induction alone, treatment of diabetic mice with propolis significantly restored the plasma cytokine and ROS levels and the lipid profile to nearly normal levels. Most importantly, compared with untreated diabetic mice, diabetic mice treated with propolis exhibited significantly enhanced lymphocyte proliferation and chemotaxis towards CCL21 and CXCL12.

**Conclusion:**

Our findings reveal the potential immuno-modulatory effects of propolis, which acts as a natural antioxidant to enhance the function of immune cells during diabetes.

## Background

Type 1 diabetes mellitus (T1D) is a chronic T-cell–mediated autoimmune disease that results in the destruction of insulin-secreting β-cells [1]. Diabetes is associated with multiple metabolic disorders that are characterized by hyperglycemia, which is accompanied by several complications [2] that result from an absolute or relative deficiency in insulin secretion or action [3]. Dyslipidemia is a common feature of diabetes, which is characterized by elevated triglyceride and low-density lipoprotein (LDL) cholesterol (LDL-C) levels [4]. Hyperglycemia or dyslipidemia easily induces extensive oxidative stress that causes serious cellular dysfunction in diabetic patients [5, 6]. Persistent hyperglycemia increases the production of free radicals, especially reactive oxygen species (ROS), in several tissues [7]. Increased lipid peroxidation, characterized by increases in the levels of malondialdehyde (MDA), results in the formation of crosslinks between single molecules in proteins and the oxidation of LDL particles; oxidized LDL serves as the most common marker of oxidative stress [8, 9].

Inflammation in autoimmune diseases is characterized by an imbalance between pro- and anti-inflammatory cytokines. Pro-inflammatory cytokines deleteriously influence insulin sensitivity and β-cell function [10]. Interestingly, altered levels of cytokines impair insulin secretion in β cells [11], and accumulating evidence supports that diabetes is a disease of the innate immune system [11, 12]. Furthermore, diabetes increases the production of pro-inflammatory cytokines, including IL-1α, IL-1β, IL-6, and CXCL10 [13, 14]. However, the main cytokines involved in diabetes pathogenesis are IL-1, TNF-α, and IL-6 [15]. The impaired production of IL-1, IL-6, TNF-α and IFN-γ and the increased production of IL-10 in type 1 diabetic peripheral blood mononuclear cell (PBMC) cultures may indicate deficiencies in mononuclear cell activation and immune cellular adaptive responses [16].

The increased incidence of infections in people with T1D is attributed to impairments in both humoral and cellular immune responses [17]. Defects in CD8^+^ CD28^+^T suppressor lymphocyte populations have been identified in patients with T1D [18]. Impairments in immune cells might interfere with normal pancreatic development and glucose homeostasis [19]. In addition, defects in lymphocyte function have been suggested to contribute to disruptions in potassium channels [20]. A previous investigation demonstrated that monocytes isolated from diabetic patients spontaneously secreted pro-inflammatory cytokines, leading to an altered T-cell response [21]. We previously reported that the decreased proliferative capacity of lymphocytes contributed to the exhaustion of T cells during T1D [22]. Chemokines play a crucial role in immune cell chemotaxis. In particular, CCL21 participates in naive T- and B-cell recruitment to the extra-follicular area in secondary lymphoid organs [23]. CCL21 and CXCL12 are produced by cells scattered throughout the extra-follicular area and act via CCR7 and CXCR4, respectively, which are specifically expressed on activated T and B cells [24]. The actin cytoskeleton is dynamically remodeled during B- and T-cell chemotaxis; this reorganization produces the force necessary for the activation and migration of these cells [25].

Diabetic complications and immune response impairment are challenges in the clinical treatment of T1D; thus, the development of more effective treatment strategies is required. Propolis is a resinous natural material produced by bees from the collected exudates and buds of plants mixed with wax and bee enzymes [26]. Propolis has several biological and pharmacological properties, such as immuno-modulatory, antitumor, anti-inflammatory, antioxidant, antibacterial and antiviral activities [27–30]. However, the mechanisms by which propolis modulates the immune system during diabetes remain poorly understood. Therefore, the current study was conducted to investigate the direct effect of propolis supplementation on the impaired function of B and T lymphocytes during T1D.

## Materials and methods

### Propolis preparation

Honey Spring propolis (batch number 4A80) was collected from Saudi Arabia by Eng. Abdullah Baqshan, Chair of Bee Research at the College of Food and Agriculture Sciences of King Saud University. Propolis was collected and characterized at our laboratory using high-speed counter current chromatography and off-line atmospheric pressure chemical ionization mass-spectrometry injection as previously described [31]. Briefly, propolis extracts were prepared in three stages: drying, extraction, and evaporation. The drying process began by washing the sample and cutting it into small pieces, which were placed in an oven at 40–60 °C for 1 hour. Prior to the extraction process, the samples were dried and then crushed using a blender. One hundred grams of dry sample were placed in a 1-L Erlenmeyer flask and soaked in 1 L of ethanol. The sample in ethanol was stirred for approximately 30 minutes and was allowed to stand overnight to settle. Then, the solution containing the active substance was filtered with filter paper. The soaking process was repeated three times. The final stage was evaporation. The extraction solvent (ethanol) was added to a 1-L evaporation flask. Then, a water bath was filled with water up to a full circuit, installed according to the manufacturer’s instructions, and set to a temperature of 90 °C. Ethanol was allowed to drip into the flask (approximately 1.5–2 hours/flask containing approximately 900 mL). The extraction yielded roughly one-tenth of the dried natural materials (10 g extract/100 g sample). The final solutions were stored in hermetically sealed brown glass bottles at room temperature (RT). Previous studies have shown that propolis extract prepared using this method is stable for 6 months, maintaining its antimicrobial and antioxidant activities over this period [32]. Abundant data from our laboratory obtained using various animal models indicate that a 50–250 mg/kg body weight daily dose of the ethanol-soluble derivative of propolis does not elicit toxic effects. Therefore, this dose is considered safe, and we used an optimal concentration (100 mg/kg body weight) of ethanol-soluble derivative of propolis for the treatment of normal and diabetic mice.

### Chemicals

Streptozotocin (STZ) was obtained from Sigma Chemicals Co. (St. Louis, MO, USA). STZ was dissolved in cold 0.01 M citrate buffer (pH 4.50), which was freshly prepared (within 5 min) as needed.

### Animals and diabetes induction

A total of 39 sexually mature 12-week-old male BALB/c mice weighing 25–30 g each were obtained from the Central Animal House of the Faculty of Pharmacy at King Saud University. All animal procedures were conducted in accordance with the standards set forth in the Guidelines for the Care and Use of Experimental Animals by the Committee for the Purpose of Control and Supervision of Experiments on Animals (CPCSEA) and the National Institutes of Health (NIH). The Animal Ethics Committee of the Zoology Department at the College of Science of King Saud University approved the protocol used in this study according to the principles of the Declaration of Helsinki. All animals were acclimated to metal cages in a well-ventilated room for 2 weeks prior to experimentation. The animals were maintained under standard laboratory conditions (23 °C, 60-70 % relative humidity and a 12-h light/dark cycle), fed a standard diet of commercial pellets and given water *ad libitum*. All mice were fasted for 20 h prior to diabetes induction. The mice (*n* = 26) were rendered diabetic via intraperitoneal (i.p.) injection of STZ (60 mg/kg body weight in 0.01 M citrate buffer, pH 4.5) daily for 5 consecutive days [22–33]; alternatively, the mice in the control group (*n* = 13) were injected with vehicle alone (0.01 M citrate buffer, pH 4.5). Three days after the final injection of STZ, the blood glucose levels were measured, and the mice were considered diabetic if the blood glucose levels exceeded 220 mg/dL. The animals were housed for 2 weeks prior to oral supplementation with propolis. The animals were divided into three experimental groups: group 1 consisted of control non-diabetic mice that received daily supplementation of 100 μL of distilled 70 % ethanol via oral gavage for one month; group 2 consisted of diabetic mice that received 100 μL of 70 % ethanol daily via oral gavage for one month; and group 3 consisted of diabetic mice that were supplemented daily with the ethanol-soluble derivative of propolis (100 mg/kg body weight) dissolved in 100 μL of 70 % ethanol via oral gavage for one month. Therefore, the volume of daily supplementation received by each mouse in the three groups was constant and did not exceed 100 μL. The optimal dose of propolis was determined in our laboratory based on its LD_50_ and several established measured parameters.

#### Sample collection

Whole blood was collected from the abdominal aorta and immediately transferred to heparinized tubes. The blood was then centrifuged at 4,000 × *g* for 10 min using a bench-top centrifuge (MSE Minor, England) to remove red blood cells and recover plasma. The plasma samples were separated, collected using dry Pasteur pipettes and stored at −80 °C until use. After plasma isolation, PBMCs were isolated using the Ficoll gradient method. Freshly isolated PBMCs were cultured in RPMI 1640 medium supplemented with 10 % fetal calf serum (FCS) and HEPES (R-10 medium) for at least 4 hours prior to the start of the experiments.

#### Blood analysis

The blood glucose levels were determined using an AccuTrend sensor (Roche Biochemicals; Mannheim, Germany). Luminex (Biotrend; Düsseldorf, Germany) was used to analyze the serum insulin levels according to the manufacturer’s instructions.

#### Measurement of the free radical levels

The levels of ROS were determined in bone marrow aspirate, spleen tissue lysate, blood and liver tissue lysate using 2,7-dichlorodihydrofluorescein diacetate (H2DCF-DA) (Beyotime Institute of Biotechnology, Haimen, China). The oxidation of 2’-7’ dichlorofluorescin (H2DCF) to 2’-7’dichlorofluorescein (DCF) has been used quite extensively for the quantitation of H2O2. The diacetate form, H2DCFDA and its acetomethyl ester H2DCFDA-AM are taken up by cells where non specific cellular esterases act upon it to cleave off the lipophilic groups, resulting in a charged compound believed to be trapped inside the cell. Oxidation of H2DCF by ROS converts the molecule to 2’, 7’ dichlorodihydrofluorescein (DCF), which is highly fluorescent. The reported wavelengths for the measurement of DCF fluorescence are 498 nm for excitation and 522 nm for emission.

#### Lipid profile analysis

The lipid profiles were determined using BioMerieux kits via a standard assay method. The cholesterol levels were evaluated using the cholesterol esterase method. High-density lipoprotein HDL, LDL-C, and chylomicrons were precipitated with phosphotungstic acid. The amount of cholesterol bound to HDL was determined using the cholesterol oxidase method and the phosphotungstate magnesium salt method using a Cholesterol E-Test Kit (Wako, Osaka, Japan).

#### Determination of the plasma cytokine levels

The plasma cytokine profiles were evaluated in triplicate using samples that had been stored at −80 °C. The plasma IFN-α level was measured using a commercial ELISA (PBL, Piscataway, NJ) according to the manufacturer’s instructions. The plasma levels of IL-1β, IL- 2, IL-4, IL-6, IL-7, IL-8, IL-10 and TNF-α were measured via ELISA using the rat Bio-Plex cytokine assay kit (Bio-Rad, Hercules, CA) according to the manufacturer’s instructions.

#### Flow cytometry

The expression of cell-surface antigens on isolated PBMCs was determined via single-parameter fluorescence-activated cell sorting (FACS) analysis using the following monoclonal antibodies (mAbs): (i) PE-conjugated anti-CD45R/B220 and PE-conjugated isotype-matched control mAbs (all purchased from R&D Systems, France) and (ii) carboxyfluorescein succinimidyl ester (CFSE, Invitrogen). A FACSCalibur flow cytometer (BD-Pharmingen) was used for data acquisition and analysis. After the gates were set to include only viable cells, 10^4^ events per sample were collected and analyzed. For each marker, the threshold for positivity was defined relative to the nonspecific binding observed in the presence of the appropriate isotype control mAb.

#### CFSE proliferation assay

Isolated PBMCs from the different groups of mice were harvested, washed twice in PBS and stained with 0.63 μM CFSE (Molecular Probes, Eugene, OR) for 8 minutes at RT. The residual CFSE was removed by three washes with PBS. The CFSE-labeled cells were seeded in 6-well plates and stimulated either with IL-4 and CD40L (for B-cell stimulation) or with 10 ng/mL staphylococcal enterotoxin B (SEB) (for T-cell stimulation); the control cells were not stimulated. The cells were then grown for 4 days in cell culture medium. After 4 days in culture, the cells were collected, stained with the PE-conjugated anti-CD45R/B220 mAb and fixed in 300 μL of 1x PBS containing 1 % formaldehyde. The CFSE fluorescence intensity was measured by flow cytometry using a FACSCalibur flow cytometer (BD-Pharmingen).

#### *In vitro* migration assay

The chemokine-dependent migration of PBMCs isolated from the different groups of mice was measured using an *in vitro* two-chamber migration assay (using Transwell plates purchased from Costar, Cambridge, MA) followed by flow cytometric analysis. Briefly, 600 μL of migration buffer alone or supplemented with CCL21 and CXCL12 (both at 500 ng/mL; R&D Systems) was added to the lower chamber, and 10^4^ cells suspended in migration buffer were added to the upper chamber. The plates were then incubated for 3 hours at 37 °C, and the input cells and the transmigrated cells were centrifuged, stained with the PE-conjugated anti-CD45R/B220 mAb, fixed in 300 μL of 1x PBS containing 1 % formaldehyde and counted for 60 seconds via flow cytometry using a FACSCalibur flow cytometer (BD-Pharmingen). The migration percentage was calculated as the percentage of input cells that migrated to the lower chamber. To calculate the change in the migration percentage induced by chemokines, the percentage of cells that migrated to the medium alone was subtracted from the percentage of cells that migrated to the medium containing the chemokines.

### Statistical analysis

The data were tested for normality (using an Anderson-Darling test) and variance homogeneity prior to further statistical analyses. The data were normally distributed and were expressed as the means ± standard error of the mean (SEM). Significant differences between groups were analyzed using one-way analysis of variance (for more than two groups) followed by Tukey’s post-test using SPSS software version 17. Differences were considered to be significant at ^*^P < 0.05 for diabetic vs. control, ^**+**^*P* < 0.05 for diabetic + propolis vs. control, or ^**#**^*P* < 0.05 for diabetic + propolis vs. diabetic.

## Results

### Characteristics of diabetic animal model and diabetes complications before and after oral supplementation with propolis

We firstly monitored changes in body weight, blood biochemical parameters and leucocyte counts in all animal groups throughout the experimental period. The treatment of mice with STZ resulted in marked decreased in the insulin level and sever hyperglycemia that was still detectable throughout the experiment period. Two weeks post STZ injection and prior to supplementation with propolis, diabetic mice exhibited a significant decrease in the body weight, leucocyte and lymphocyte counts compared to control non diabetic animals (*P < 0.05) (Table 1). Additionally, diabetic mice exhibited a significant increase in levels of ROS, IL-6, cholesterol and creatinine compared to control non diabetic animals (*P < 0.05). Then the diabetic mice were randomly distributed into two groups: group 2 consisted of diabetic mice that received 100 μL of 70 % ethanol (vehicle) daily via oral gavage for one month; and group 3 consisted of diabetic mice that were supplemented daily with the ethanol-soluble derivative of propolis (100 mg/kg body weight) dissolved in 100 μL of 70 % ethanol via oral gavage for one month.

**Table 1:** Influence of diabetes induction by STZ and propolis supplementation to diabetic mice on the body weight and blood biochemical parameters

Days post STZ or vehicle injection	Groups	Body weight	Glucose	Insulin	ROS	IL-6	Cholesterol	Creatinine	WBC count	Lymphocyte count
		(g)	(mg/dl)	(ng/ml)	(nmol/ml)	(pg/ml)	(mg/100 ml)	(dg/ml)	(x10^3^/mm^3^)	(x10^3^/mm^3^)
3Day 3	Control	28.8 ± 1.9	103 ± 11	6.6 ± 0.48	33 ± 2.8	19 ± 2.4	37 ± 2.8	5.2 ± 0.44	15 ± 1.4	10.6 ± 1.2
	Diabetic	29 ± 1.7	243 ± 21.4*	4 ± 0.35*	42 ± 4.6*	28.4 ± 3.1*	35.8 ± 3.2	5.4 ± 0.52	12.4 ± 1.1*	8 ± 0.68*
Day 14	Control	30 ± 2.3	93 ± 8.2	6.4 ± 0.61	36 ± 3.4	18 ± 2.2	38.4 ± 2.4	4.8 ± 0.6	15.4 ± 1.6	10.4 ± 1.6
	Diabetic	25 ± 2.1*	297 ± 24.6*	2.8 ± 0.3*	77 ± 5.8*	46 ± 4.2*	53 ± 4.2*	7.8 ± 0.62*	11 ± 1.2*	7.4 ± 0.8*
Weeks post propolisor vehicle treatment	Groups									
Week 1	Control	32 ± 2.4	109 ± 8.8	5.7 ± 0.5	27.1 ± 2.9	24.6 ± 2.4	33 ± 3.2	5.4 ± 0.5	15.8 ± 1.1	10.7 ± 1.1
	Diabetic	24.6 ± 2.1*	374 ± 31.2*	3.3 ± 0.4*	79.8 ± 5.5*	44 ± 5.2*	62 ± 5.4*	7.9 ± 0.22*	12 ± 1.2*	7.8 ± 0.9*
	Diab + Propolis	26.8 ± 2.4^+^	287 ± 24.8^#^^+^	4.2 ± 0.44^+^	44.1 ± 4.2^#^^+^	41 ± 4.2^+^	58.4 ± 5.8^+^	7.7 ± 0.3^+^	12.7 ± 1.6^+^	9.1 ± 4.1^#^^+^
Week 2	Control	33.4 ± 3.6	96 ± 10.4	7.1 ± 0.75	39 ± 5.4	22 ± 2.7	39 ± 4.2	5.3 ± 0.75	15.4 ± 0.88	10.8 ± 1.2
	Diabetic	23.6 ± 3.1*	411 ± 34.6*	2.6 ± 0.29*	98.6 ± 8.4*	66 ± 5.2*	79 ± 6.4*	8.2 ± 0.9*	11 ± 0.9*	7.6 ± 0.9 *
	Diab + Propolis	28.4 ± 2.4^#^^+^	284 ± 26^#^^+^	3.9 ± 0.38^#^^+^	64 ± 4.8^#^^+^	34 ± 3.2^#^^+^	61.2 ± 5.5^#^^+^	5.9 ± 0.48^#^	12.4 ± 0.5^#^^+^	9.1 ± 0.92^+^
Week 3	Control	34.2 ± 4.2	89 ± 11.4	5.8 ± 0.6	25.5 ± 3.2	26 ± 2.4	22.8 ± 3	4.8 ± 0.6	15.8 ± 1.22	10.9 ± 1.1
	Diabetic	23 ± 2.8*	382 ± 31*	2.2 ± 0.2*	102 ± 9.2*	68.8 ± 3.2*	82 ± 8.4*	8.46 ± 0.8*	8.4 ± 0.8 *	7.1 ± 0.6 *
	Diab + Propolis	28.8 ± 3.5^#^^+^	261 ± 25.5^+^	3.5 ± 0.34^#^^+^	51.6 ± 4.6^#^^+^	40 ± 3.8^#^^+^	42.3 ± 5.5^#^^+^	6.22 ± 0.44^#^^+^	13.1 ± 1.42^#^^+^	10.2 ± 0.65^#^^+^
Week 4	Control	36.6 ± 2.9	119 ± 14	5.2 ± 0.45	31.5 ± 4.1	23 ± 3.4	19 ± 2.2	4.7 ± 0.42	15.4 ± 1.2	10.8 ± 1.4
	Diabetic	22.84 ± 2.8*	368 ± 22*	1.8 ± 0.2*	144 ± 11.2*	79 ± 9*	59.6 ± 5.4*	8.8 ± 0.9*	8.5 ± 0.8*	6.7 ± 0.8*
	Diab + Propolis	29.2 ± 2.6^#^^+^	244 ± 18^#^^+^	3.4 ± 0.35^#^^+^	48.6 ± 5.6^#^^+^	49 ± 6^#^^+^	37 ± 3.2^#^^+^	5.99 ± 0.37^#^^+^	14 ± 0.18^#^	10.1 ± 0.96^#^

The body weight and blood biochemical parameters were measured in the 3 groups of mice throughout the experiment period. The pooled data for 3 mice from each group are expressed as the mean value for each parameter ± SEM

*P < 0.05 for diabetic vs. control

^#^ *P* < 0.05 for diabetic + propolis vs. diabetic

^+^ *P* < 0.05 for diabetic + propolis versus control (ANOVA followed by Tukey’s post-test)

Treatment of diabetic mice with propolis for 4 weeks had a clear and significant (^#^*P* < 0.05) ameliorative effect on the body weight and all the blood biochemical parameters when compared to diabetic mice that were supplemented with vehicle.

### Modulation of the plasma cytokine levels in diabetic mice supplemented with propolis

We then monitored the blood glucose and insulin levels in the three groups of animals at the end of the experiment period and found that the induction of diabetes in mice by STZ was associated with a significant elevation in the blood glucose level, a marked reduction in the circulating lymphocyte count and an evident decrease in the insulin levels compared to the control treatment (*P < 0.05, n = 10) (Table 2). The oral supplementation of diabetic mice with the ethanol-soluble derivative of propolis significantly increased the circulating lymphocytes count compared to diabetes induction alone (^#^*P* < 0.05, *n* = 10). Although the propolis-treated diabetic mice displayed high glucose levels, they exhibited a significant decrease in their blood glucose level compared with diabetic mice, and their insulin levels were restored (^#^*P* < 0.05). We also monitored the plasma cytokine levels in the 3 experimental groups because these levels affect the normal function of immune cells. The accumulated data from 10 individual mice from each group are shown in Table 2. The diabetic mice exhibited aberrant and significantly elevated levels of pro-inflammatory cytokines (IL-1β, IL-6 and TNF-α) and markedly reduced levels of IL-2, IL-4 and IL-7 compared with the control non-diabetic mice (*P < 0.05). Interestingly, treatment of diabetic mice with the ethanol-soluble derivative of propolis significantly (^#^*P* < 0.05) restored the levels of these plasma mediators to nearly normal levels compared with diabetes induction alone. In contrast, neither the induction of diabetes nor supplementation with propolis affected the plasma levels of IL-8 or IL-10.

**Table 2:** Effects of propolis administration to diabetic mice on the plasma levels of glucose, insulin and cytokines

Parameters	Control mice	Diabetic mice	Diabetic mice supplemented with propolis
Blood glucose (mg/dl)	119 ± 14	368 ± 22*	244 ± 18^#^^+^
Insulin (ng/ml)	5.2 ± 0.45	1.8 ± 0.2*	3.4 ± 0.35^#^^+^
WBCs count (10^3^/μl)	15.4 ± 1.2	8.5 ± 0.8*	14 ± 0.18^#^
Lymphocytes (%)	77 ± 6.5	49 ± 5*	72 ± 7.4^#^
Monocytes (%)	5 ± 0.8	5.1 ± 0.5	4.9 ± 0.75
Neutrophils (%)	21.4 ± 3.1	21.5 ± 3.4	22 ± 2.8
IL-1 β (pg/ml)	37 ± 4	144 ± 12*	78 ± 9.2^#^^+^
IL-6 (pg/ml)	23 ± 3.4	79 ± 9*	49 ± 6^#^^+^
TNF-α (pg/ml)	17 ± 2.2	64 ± 8.2*	42 ± 4.8^#^^+^
IL-2 (pg/ml)	111 ± 9.6	44 ± 7*	101 ± 9.2^#^
IL-7 (pg/ml)	129 ± 11	34 ± 4.8*	119 ± 10^#^
IL-4 (pg/ml)	44 ± 5.5	11 ± 1.5*	43 ± 4.9^#^
IL-8 (pg/ml)	66 ± 8.5	69 ± 7.6	70 ± 7.8
IL-10 (pg/ml)	84 ± 9.4	78.6 ± 8.2	86 ± 9.5

The plasma levels of glucose, insulin and cytokines including IL-1β, IL-2, IL-4, IL-6, IL-7, IL-8, IL-10 and TNF-α were measured in the 3 groups of mice at the end of the experiments. The pooled data for 10 mice from each group are expressed as the mean value for each parameter ± SEM

^*^ *P* < 0.05 for diabetic vs. control

^#^ *P* < 0.05 for diabetic + propolis vs. diabetic

^**+**^ *P* < 0.05 for diabetic + propolis versus control (ANOVA followed by Tukey’s post-test)

### Treatment of diabetic mice with propolis decreased the levels of free radicals in different organs

The ROS levels were detected in the plasma and in tissue lysates of the bone marrow (the primary lymphoid organ and the origin of all immune cells), the spleen (a secondary lymphoid organ that is a site of antigen recognition), and the liver. The accumulated data from 10 individual mice from each group are shown in Fig. 1. The ROS levels of the diabetic mice were significantly higher than those of the control mice (*P < 0.05). Oral supplementation of the diabetic mice with the ethanol-soluble derivative of propolis significantly restored the levels of ROS close to the level of control mice when compared to diabetes induction alone (^#^*P* < 0.05).

**Fig. 1:** Significant alterations in the levels of ROS in different organs of diabetic mice after supplementation with propolis. The levels of ROS were determined in control mice (open bars), diabetic mice (black bars) and propolis-treated diabetic mice (hatched bars) as described in the Materials and Methods section. The pooled data for 10 mice from each group are expressed as the mean ROS level ± SEM. ^*^ *P* < 0.05 for diabetic versus control; ^#^ *P* < 0.05 for diabetic + propolis versus diabetic; ^+^ *P* < 0.05 for diabetic + propolis versus control (ANOVA followed by Tukey’s post-test)

### Diabetic mice exhibit markedly changed lipid profiles, displaying a tendency toward abnormal obesity

The induction of diabetes is commonly associated with dyslipidemia, a phenomenon characterized by altered plasma lipid profiles and an increased risk of cardiovascular disease. Therefore, we monitored the lipid profiles in the 3 groups of animals. The accumulated data from 10 individual mice from each group are shown in Fig. 2. The LDL-C and total cholesterol levels were significantly higher in plasma of the diabetic mice than in that of the control non-diabetic mice (*P < 0.05). Similarly, the levels of MDA (a marker of oxidative lipid damage and a major oxidative product of peroxidized polyunsaturated fatty acids) were significantly higher in plasma of the diabetic mice than in that of the control non-diabetic mice (*P < 0.05). In contrast, the level of HDL-C was significantly lower in plasma of the diabetic mice than in that of the control non-diabetic mice (*P < 0.05). Supplementation of the diabetic mice with the ethanol-soluble derivative of propolis significantly restored the plasma lipid profiles to nearly normal levels compared to diabetes induction alone (^#^*P* < 0.05).

**Fig. 2:** Propolis restores the lipid profile in diabetic mice. The levels of HDL-C, LDL-C, total cholesterol and MDA were determined in control mice (open bars), diabetic mice (black bars) and diabetic mice supplemented with propolis (hatched bars) as described in the Materials and Methods section. The pooled data for 10 mice from each group are expressed as the mean level of each lipid ± SEM. ^*^ *P* < 0.05 for diabetic versus control; ^**#**^ *P* < 0.05 for diabetic + propolis versus diabetic; ^**+**^ *P* < 0.05 for diabetic + propolis versus control (ANOVA followed by Tukey’s post-test)

### Treatment of diabetic mice with propolis enhances antigen stimulation and the proliferation of B and T lymphocytes

Because decreased levels of IL-2 and IL-7 may result in reduced lymphocyte proliferation, we examined the levels of B and T lymphocytes using a CFSE dilution assay in the diabetic mice after antigen stimulation. PBMCs were isolated from the three groups of mice, and these cells were then labeled with CFSE. The CFSE-labeled cells were stimulated either with SEB or with IL-4 and CD40L; alternatively, the control cells were not stimulated. The cells were then grown for 4 days in cell culture medium. After 4 days in culture, the cells were stained with a PE-CD45R/B220 mAb, and their proliferative capacity was analyzed using flow cytometry. The plots were first gated for lymphocytes according to forward and side scatter and then for viable cells to exclude dead cells. One representative experiment is shown to demonstrate the method used to analyze CFSE-stained B cells (after gating for viable lymphocytes and then gating for the CD45R+/B220+ population) (Fig. 3a). The percentage of proliferating cells (CFSE-lo) in the 3 experimental animal groups is indicated in each panel. The percentage of proliferating B cells following IL-4 and CD40L stimulation increased from 3 % to 86 % (83 % specific proliferation) in the control non-diabetic mice, from 5 % to 31 % (26 % specific proliferation) in the diabetic mice and from 4 % to 80 % (76 % specific proliferation) in the diabetic mice treated with the ethanol-soluble derivative of propolis (Fig. 3b). Accumulated data from 10 separate experiments in each group revealed that stimulation with IL-4 and CD40L significantly reduced the percentage of proliferating B lymphocytes by 3-fold in the diabetic group relative to the control group (*P < 0.05). Interestingly, the percentage of proliferating B lymphocytes was significantly (^#^*P* < 0.05) restored in the propolis-treated diabetic group compared with the untreated diabetic group (Fig. 3c). Similarly, accumulated data from 10 experiments from each group demonstrated that the percentage of proliferating T lymphocytes (CD45R/B220^neg^ population) was significantly (*P < 0.05) decreased in the diabetic mice compared with the control mice (Fig. 3d). The diabetic mice exhibited a significant restoration in the percentage of proliferating T lymphocytes following treatment with the ethanol-soluble derivative of propolis compared with the untreated diabetic mice (^#^*P* < 0.05).

**Fig. 3:** Altered proliferative capacity of B and T lymphocytes in diabetic mice supplemented with propolis. The proliferative capacity of B lymphocytes in response to stimulation with IL-4 and CD40L and of T lymphocytes in response to stimulation with SEB was evaluated using CFSE assays and flow cytometry. **a** Representative dot plots showing the gating strategy to obtain viable lymphocytes based on forward and side scatter and to discriminate between the CD45R/B220^+^ cell population (B-lymphocytes) and the CD45R/B220^neg^ cell population (T-lymphocytes) using an CD45R/B220-PE mAb and flow cytometric analysis. **b** One representative experiment showing the analysis of CFSE-stained B cells (after gating for viable cells); the percentage of proliferating cells (CFSE-lo) in control, diabetic and propolis-treated diabetic mice is indicated in each panel. **c** & **d** The data from the different experiments (n = 10) are expressed as the mean percentage of proliferating cells ± SEM in response to stimulation either with IL-4 and CD40L or with SEB in control mice (open bars), diabetic mice (black bars), or propolis-treated diabetic mice (hatched bars). ^*^ *P* < 0.05 for diabetic versus control; ^**#**^ *P* < 0.05 for diabetic + propolis versus diabetic; ^**+**^ *P* < 0.05 for diabetic + propolis versus control (ANOVA followed by Tukey’s post-test)

### Supplementation of diabetic mice with propolis enhances CCL21- and CXCL12-mediated chemotaxis in B and T lymphocytes

CCL21 and CXCL12 play essential roles in the trafficking and homing of B and T cells to lymphoid tissues and in subsequent antigen recognition. We assessed the chemotactic response of B and T lymphocytes toward CCL21 and CXCL12 using a chemotaxis assay and flow cytometric analysis. The plots were first gated for lymphocytes according to forward and side scatter and then for viable cells to exclude dead cells. The input cells and the PBMCs that migrated to medium alone or medium supplemented with chemokines were stained with PE-CD45R/B220 (Fig. 4a). In one representative experiment, the percentage of migrated PE-CD45R/B220^positive^ B cells increased from 2 % in medium alone to 50 % in CCL21-containing medium (48 % specific migration) and to 66 % in CXCL12-containing medium (64 % specific migration) in the control mice, from 3 % in medium alone to 22 % in CCL21-containing medium (19 % specific migration) and to 29 % in CXCL12-containing medium (26 % specific migration) in the diabetic mice and from 1 % in medium alone to 33 % in CCL21-containing medium (32 % specific migration) and to 50 % in CXCL12-containing medium (49 % specific migration) in the diabetic mice treated with the ethanol-soluble derivative of propolis (Fig. 4A). Similarly, the percentage of migrated PE-CD45R/B220^neg^ T cells increased from 1 % in medium alone to 59 % in CCL21-containing medium (58 % specific migration) and to 78 % in CXCL12-containing medium (77 % specific migration) in the control mice, from 2 % in medium alone to 24 % in CCL21-containing medium (22 % specific migration) and to 33 % in CXCL12-containing medium (31 % specific migration) in the diabetic mice and from 1 % in medium alone to 52 % in CCL21-containing medium (51 % specific migration) and to 72 % in CXCL12-containing medium (71 % specific migration) in the diabetic mice treated with the ethanol-soluble derivative of propolis. Accumulated data from 10 experiments from each group are expressed as the mean percentage of chemokine-mediated specific migration of B and T lymphocytes ± SEM (Fig. 4b & c). The percentage of specific B- and T-lymphocyte migration in response to CCL21 and CXCL12 was significantly decreased in the diabetic group compared with the control group (*P < 0.05). Interestingly, the percentage of specific B- and T-lymphocyte migration in response to CCL21 and CXCL12 was significantly (^#^*P* < 0.05) restored in the propolis-treated diabetic group compared with the untreated diabetic group.

**Fig. 4:** Modulation of chemokine-mediated chemotaxis by B and T lymphocytes from propolis-treated diabetic mice. PBMCs were subjected to migration assays in response to CCL21 and CXCL12. **a** Representative dot plots showing the gating strategy to obtain viable lymphocytes based on forward and side scatter and to discriminate between the CD45R/B220^+^ cell population (B-lymphocytes) and the CD45R/B220^neg^ cell population (T-lymphocytes) using a PE-CD45R/B220 mAb and flow cytometric analysis. The input cells and the migrated cells were stained with the PE-CD45R/B220 mAb. The cells were then counted for 60 seconds via flow cytometry to calculate the percentage of cells that migrated nonspecifically (based on the number of cells that migrated to medium alone) or specifically (based on the number of cells that migrated to medium containing a chemokine). To calculate the percentage of specific migration induced by chemokines, the percentage of cells migrating to medium alone was subtracted from the percentage of cells migrating to the medium containing a chemokine. **b** & **c** The data from the different experiments (n = 10) are expressed as the mean percentage of chemokine-mediated specific migration of B and T lymphocytes ± SEM in control mice (open bars), diabetic mice (black bars) or propolis-treated diabetic mice (hatched bars). ^*^ *P* < 0.05 for diabetic versus control; ^**#**^ *P* < 0.05 for diabetic + propolis versus diabetic; ^**+**^ *P* < 0.05 for diabetic + propolis versus control (ANOVA followed by Tukey’s post-test)

## Discussion

Natural antioxidants play central roles in enhancing the immune system via mechanisms that depend on oxidative stress; in turn, oxidative stress appears to play significant roles in many human diseases. In this context, we previously demonstrated that thymoquinone benefits the treatment of multiple myeloma and alleviates diabetic complications by restoring the T-cell immune response in diabetic offspring [34–36]. Interestingly, we showed that natural antioxidants isolated from snake and ant venoms were able to enhance normal lymphocyte function and exert antitumor effects on breast cancer cells [37, 38]. Propolis is a natural antioxidant product found in plant materials and is processed by worker bees. Natural antioxidants play various biological roles in the treatment of diabetic complications, including impaired wound healing [39–41] and T-cell immune responses, in offspring born to diabetic mothers, as well as the treatment of other diseases, including cancer [42–44]. Cytokines are essential mediators of intercellular communication that orchestrate the interactions of immune cells during immune responses. Thus, cytokine imbalances play a significant role in the acceleration of lupus-like autoimmune disease. Our study showed that oral supplementation of diabetic mice with propolis modulated glycemia by decreasing the blood glucose levels and increasing the insulin level to values similar to those observed in non-diabetic control mice. Moreover, treating diabetic mice with propolis improved the lipid profile and significantly inhibited oxidative stress by reducing lipid peroxidation and the free ROS levels in blood and in the liver and lymphoid organs. These improvements suggested that propolis acted as a strong anti-oxidant to ameliorate oxidative stress and delay the occurrence of diabetic complications. Our data are consistent with the results of a previous study, which reported that propolis significantly increased the plasma level of insulin [45]. Furthermore, Fuliang et al. [46] observed that the administration of propolis to STZ-induced diabetic rats may control glycemia and modulate glucose and lipid metabolism, leading to decreased release of lipid peroxidation products and increased free radical scavenging in diabetic rats.

Moreover, the oral administration of propolis extract significantly suppressed the blood glucose levels and helped to reduce dyslipidemia in diabetic rats [47]. Propolis, which displays strong anti-oxidant activity, has been confirmed to suppress the MDA level and increase anti-oxidant activity in diabetic animal models and human patients [48–50]. Diabetic complications are primarily attributed to increased ROS levels due to hyperglycemia [51, 52]. Clinical trials also showed that improving oxidative stress may prevent the progression of both types of diabetes [53, 54].

Importantly, T1D contributes to prolonged inflammation, which is characterized by the impairment of the immune response due to elevated levels of IL-1β, IL-6, and TNF-α [55, 56]. Therefore, targeting inflammatory mediators has been proposed as an effective strategy to improve the immune response and modulate inflammation in diabetic patients. In the present study, we showed that propolis supplementation abrogated the inflammatory process associated with diabetes and restored the levels of IL-1 β, IL-6 and TNF-α to nearly normal levels. Propolis has been shown to directly inhibit cytokine production by immune cells [57]. Khayyal et al. (2003) showed that the administration of an aqueous extract of propolis for the treatment inflammatory diseases decreased the levels of pro-inflammatory cytokines (TNF-α and IL-6) [58].

In the present study, the plasma levels of IL-2, IL-4 and IL-7 were significantly reduced in diabetic mice, providing important evidence of impaired immune function. However, the IL-8 and IL-10 levels did not differ between diabetic mice and control mice or propolis-treated diabetic mice in this study. Furthermore, the plasma levels of IL-2, IL-4 and IL-7 were markedly decreased in diabetic mice, and these decreases were accompanied by a marked reduction in the proliferative capacity of antigen-stimulated B and T lymphocytes. Several studies have revealed that the plasma levels of IL-2, which promotes T-lymphocyte survival and proliferation, are consistently decreased in several diseases, indicating defective T-cell function. Furthermore, IL-7 plays complimentary roles in the maintenance of T cells after antigen stimulation [59]. T cell survival may be impaired in the absence of IL-7 [60]. Notably, the acute homeostatic proliferation of memory T cells has been shown to partly depend on the endogenous IL-7 levels [61]. Additionally, IL-7 plays several important roles during B-cell development, including promoting the proliferation and survival of B-cell progenitors and the maturation of B cells during the pro-B- to pre-B-cell transition [62]. Impaired T- and B-lymphocyte function has been linked to the abnormal activation of the immune system and has been shown to contribute to immunodeficiency [63, 64]. In this study, we found that treating diabetic mice with propolis significantly restored both the levels of IL-2 and IL-7 and the proliferation of B and T lymphocytes. This restorative effect of propolis enhanced and maintained an efficient immune response by lymphocytes during T1D.

Chemokines play a crucial role in immune cell chemotaxis. CXCL12 and CCL21 participate in naive T- and B-cell recruitment to the extra-follicular area in secondary lymphoid organs via their lymphocyte receptors [65]. Chemotaxis is an essential phenomenon for evaluating immune responses, and blocking chemokine receptors has recently been identified as a therapeutic strategy for various inflammatory and autoimmune diseases. Our data demonstrated that the percentages of chemotactic B and T cells were significantly reduced in diabetic mice but that treatment of diabetic mice with propolis significantly increased the percentages of chemotactic B and T cells. Supporting our results, previous studies reported that CD34+ cells isolated from diabetic patients demonstrated a marked defect in migration toward CXCL12 [66]. Moreover, the CXCR4/CXCL12 signaling pathway has been shown to protect non-obese diabetic mice from autoimmune diabetes [67]. Our results showed for the first time that propolis supplementation increased CCL21- and CXCL12-mediated B- and T-cell chemotaxis in diabetic mice. Previous studies have shown that CCR7 and CXCR4 are involved in the recruitment of blood-borne leukocytes to sites of inflammation [68]. CCL21 and its lymphocyte receptor (CCR7) play a key role in the migration of lymphocytes from blood into lymphoid tissues [69–71]. Recently, propolis has been shown to influence the immune system [72, 73]. The immuno-modulatory activity of propolis has been shown to enhance innate immunity by activating the initial steps of the immune response via the upregulation of TLR-2 and TLR-4 expression, thereby contributing to lymphocyte activation by antigen-presenting cells [73].

## Conclusions

Our data suggest that treatment with propolis enhanced B- and T-cell chemotaxis efficiency in diabetic mice. Taken together, our data suggest that propolis attenuates abnormal lipid profiles, oxidative stress, inflammation, and impaired lymphocyte proliferation and migration towards chemokines to maintain an efficient lymphocyte immune response. Therefore, the use of propolis is a potential strategy for the treatment of diabetic complications.

## Abbreviations

CFSE: Carboxyfluorescein succinimidyl ester
CCL21: CC chemokine ligand 21
CXCL12: CXC chemokine ligand 12
DM: Diabetes mellitus
HDL: High-density lipoprotein
IL: Interleukin
LDL: Low-density lipoprotein
MDA: Malondialdehyde
PBMCs: Peripheral blood mononuclear cells
ROS: Reactive oxygen species
STZ: Streptozotocin
TNF-α: Tumor necrosis factor-alpha
